The article "Supramolecular Self-Assembled Peptide-Based Vaccines: Current State and Future Perspectives" was published in 2020. Journal: Front Chem.

# Supramolecular Self-Assembled Peptide-Based Vaccines: Current State and Future Perspectives

**DOI:** 10.3389/fchem.2020.598160

**Published:** 2020-10-30

**Authors:** Turdimuhammad Abdullah, Khushbu Bhatt, Loek J. Eggermont, Nick O'Hare, Adnan Memic, Sidi A. Bencherif

**Affiliations:** ^1^Center of Nanotechnology, King Abdulaziz University, Jeddah, Saudi Arabia; ^2^Department of Pharmaceutical Sciences, Northeastern University, Boston, MA, United States; ^3^Department of Chemical Engineering, Northeastern University, Boston, MA, United States; ^4^Department of Bioengineering, Northeastern University, Boston, MA, United States; ^5^Harvard John A. Paulson School of Engineering and Applied Sciences, Harvard University, Cambridge, MA, United States; ^6^Sorbonne University, UTC CNRS UMR 7338, Biomechanics and Bioengineering (BMBI), University of Technology of Compiègne, Compiègne, France

**Keywords:** supramolecular, peptides, self-assembly, vaccine, delivery

## Abstract

Despite the undeniable success of vaccination programs in preventing diseases, effective vaccines against several life-threatening infectious pathogens such as human immunodeficiency virus are still unavailable. Vaccines are designed to boost the body's natural ability to protect itself against foreign pathogens. To enhance vaccine-based immunotherapies to combat infections, cancer, and other conditions, biomaterials have been harnessed to improve vaccine safety and efficacy. Recently, peptides engineered to self-assemble into specific nanoarchitectures have shown great potential as advanced biomaterials for vaccine development. These supramolecular nanostructures (i.e., composed of many peptides) can be programmed to organize into various forms, including nanofibers, nanotubes, nanoribbons, and hydrogels. Additionally, they have been designed to be responsive upon exposure to various external stimuli, providing new innovations in the development of smart materials for vaccine delivery and immunostimulation. Specifically, self-assembled peptides can provide cell adhesion sites, epitope recognition, and antigen presentation, depending on their biochemical and structural characteristics. Furthermore, they have been tailored to form exquisite nanostructures that provide improved enzymatic stability and biocompatibility, in addition to the controlled release and targeted delivery of immunomodulatory factors (e.g., adjuvants). In this mini review, we first describe the different types of self-assembled peptides and resulting nanostructures that have recently been investigated. Then, we discuss the recent progress and development trends of self-assembled peptide-based vaccines, their challenges, and clinical translatability, as well as their future perspectives.

The article "Supramolecular Self-Assembled Peptide-Based Vaccines: Current State and Future Perspectives" was published in 2020. Journal: Front Chem.

## Introduction

Vaccination has been considered as one of the crowning achievements of humankind, and gained remarkable triumph in treating many life-threatening and epidemic diseases, such as influenza, tuberculosis, and smallpox (Malonis et al., 2019; Piot et al., 2019). Vaccines can greatly reduce the burden of preventable infectious diseases by working with the body's natural defenses to safely develop immunity to diseases (Piot et al., 2019; Parvizpour et al., 2020). For instance, to respond to the new and unprecedented coronavirus disease 2019 (COVID-19) crisis, vaccination is considered to be the best strategy to end this pandemic (Graham, 2020; Lurie et al., 2020). Conventional vaccination methods are based on pathogens (e.g., attenuated, inactivated, toxins, subunits) that can provoke immunity against antigens and provide long-lasting protection against the diseases (Chiang et al., 2010; Cockburn and Seder, 2018). Despite these advantages, this approach is suffering from a number of drawbacks, including low immunogenicity, high cost, manufacturing challenges, vaccine instability in the cold chain, and potential contaminations during manufacturing which could alter vaccine efficacy and cause a strong allergic shock (Skwarczynski and Toth, 2016).

Although great advances have been made in the development of vaccines and immunotherapies, there is an increasing demand for enhanced control over the immune responses induced against infectious diseases and cancer. Biomaterials can be leveraged for modulating the immune system and subsequently controlling immune responses (Bookstaver et al., 2018). For instance, recent immunization strategies have centered on biomaterial-based vaccines in which specific cellular components were used as antigens to stimulate the immune response against cancer (Bencherif et al., 2015; Malonis et al., 2019). Within these biomaterial-based vaccines, full-length proteins, and peptides have been extensively studied as antigens, but they can also be used as structural biomaterials (Skwarczynski and Toth, 2016). Peptides are biomolecules that generally consist of sequences of 2-50 amino acids and that have a molecular structure that is generally much simpler than that of proteins (Malonis et al., 2019). Using peptides has become a widespread trend in vaccine development since they are easily processed and presented by antigen-presenting cells, leading to potent T-cell-mediated immune responses (Purcell et al., 2007). Furthermore, current challenges associated with cell-based or protein-based vaccination, such as manufacturing complexity, biological contamination, off-target effects, and autoimmunity, can be prevented with peptide-based vaccines (Purcell et al., 2007; Skwarczynski and Toth, 2016). Additionally, peptides are capable of self-assembly into ordered supramolecular structures, making them excellent building blocks to form nanofibers, nanovesicles, nanotubes, nanomicelles, and hydrogels (Habibi et al., 2016; Qi et al., 2018). These peptide assemblies can have a multivalent character and present peptides in their native 3D conformation, which is essential for B-cell stimulation. Furthermore, they allow mixing of multiple components with precise stoichiometry (Wen and Collier, 2015). Ultimately, immunogenic, long-lasting, stable, and self-adjuvanted vaccines can be engineered by combining epitopes, antigens, and immunomodulatory moieties within the self-assembled peptide structures (Wen and Collier, 2015).

The article "Supramolecular Self-Assembled Peptide-Based Vaccines: Current State and Future Perspectives" was published in 2020. Journal: Front Chem.

Besides being exploited as immunostimulatory materials in vaccine development, self-assembled supramolecular peptides are also excellent candidates to serve as carriers for the delivery of immunological factors (Sis and Webber, 2019; Xiao et al., 2019b). The macrostructural features of supramolecular peptide assemblies can be fine-tuned by altering the amino acid sequences. Additionally, bioactive segments can be introduced into the peptides during their self-assembly to design stimuli-responsive and cell- or organ-targeted vaccine delivery vehicles (Sis and Webber, 2019; Xiao et al., 2019a; Lampel, 2020). Moreover, combining immunogenic peptide epitopes with non-immunogenic peptides that form delivery carriers could enhance vaccine efficacy while reducing unwanted side effects (Eskandari et al., 2017).

In this mini review, we first describe the various strategies employed to create self-assembled supramolecular peptides with sophisticated hierarchical nanostructures. Next, their application in subunit vaccine design and delivery for cellular and humoral immunity is highlighted. Finally, we discuss the challenges and clinical translatability of self-assembled peptide-based vaccines, as well as their future perspectives.

## Design of Supramolecular Self-Assembled Peptides

Molecular self-assembly is a bottom-up approach for achieving highly ordered and stable nanoscale structures or patterns. This technique is based on the spontaneous assembly of small molecules or nanosized building blocks under thermodynamic equilibrium conditions (Qi et al., 2018). Intermolecular and intramolecular interactions, such as hydrogen bonding, amphiphilic interactions, and aromatic stacking, have been used for supramolecular peptide assembly, allowing the construction of complexes with stratified nanostructures (Lampel, 2020). Specifically, peptides can be designed to exhibit distinctive secondary structures, such as β-sheets, β-hairpins, and α-helices, and these natural motifs can be leveraged to drive a complex hierarchical architecture (Rad-Malekshahi et al., 2015). For instance, β-sheets consisting of alternating hydrophobic and hydrophilic amino acids have been extensively applied in driving self-assembly of peptides into extended fibrillar nanostructures (Moore et al., 2018; Sis and Webber, 2019). Several groups have designed self-assembled nanofibrils from the synthetic amphiphilic peptide RADA16 (RADARADARADARADA) through the β-sheet motifs (Figure 1A), in which alternating regions of hydrophobic alanine and hydrophilic arginine/aspartate residues can yield a stable β-sheet-rich structure (Cormier et al., 2013; Lu et al., 2019). Furthermore, the antiparallel orientation of double-layered β-sheets, such as β-hairpins, have shown to generate another secondary structure, which promotes the formation of peptide-based nanofibrous hydrogels under physiological conditions (Worthington et al., 2017). Smith et al. developed a multiphase transitioning, injectable hydrogel through the molecular self-assembly of a peptide-based β-hairpin. Their anastomosis photocage 1 (APC1) peptide, which contains seven lysine residues, was folded into a β-hairpin and rapidly self-assembled into a cross-linked fibrillar hydrogel (Smith et al., 2016). Alternatively, α-helices could also be used to form a highly ordered structure through helical self-assembly, which closely resembles the sophisticated hierarchical coiled coil-type structures of native proteins, such as collagen (Lampel, 2020). Thomson et al. designed supercoiled coil α-helical barrels by self-assembling 5-7 α-helices twisted around each other with cyclic or dihedral symmetry (Figure 1B). The peptides used in their study have a canonical hpphppp heptad repeat sequence, in which h and p represent hydrophobic and polar amino acids, respectively (Thomson et al., 2014; Rhys et al., 2018). Di-phenylalanine peptide (FF) is another interesting building block to trigger peptide self-assembly into desirable nanostructures such as nanotubes, nanospheres, and nanoribbons (Habibi et al., 2016). While self-assembly of the FF motif is usually achieved in the form of amyloid-like sheets (Lampel, 2020), Bera et al. interestingly generated a helical architecture by simply adding one more amino acid (proline) to the FF peptide, forming proline-phenylalanine-phenylalanine (PFF) (Bera et al., 2019).

The article "Supramolecular Self-Assembled Peptide-Based Vaccines: Current State and Future Perspectives" was published in 2020. Journal: Front Chem.

**Figure 1:** Strategies to induce supramolecular self-assembly of peptides and peptide-based vaccines. **(A)** Formation of β-strands from self-assembling peptide RADA16-I (top) and their arrangement into nanofibers with different symmetry classes arranged into stacks of two β-sheets (bottom). β-sheets are formed by alternating segments of hydrophobic alanine (green) and hydrophilic arginine/aspartate (blue/red) regions (reproduced with permission from Cormier et al., 2013). **(B)** Symmetry (top) and sequence (bottom) of coiled-coils (CCs) made of peptides containing a heptad repeat of hydrophobic (h) and polar (p) residues in a hpphppp pattern. Helical wheels for classical Type-N, and Type-1, Type-2, and Type-3 interfaces are depicted. All are viewed along the α-helices from the N to C termini, labels are for the canonical a–g nomenclature and the teardrop shapes indicate the direction of Cα-Cβ bonds (reproduced with permission from Rhys et al., 2018). **(C)** Effect of different divalent transition metal ions on the morphological transformation of self-assembled PAs, consisting of hexahistidine as a hydrophilic head and oligostyrene as a hydrophobic tail (reproduced from Knight et al., 2018). **(D)** Schematic illustration of immune stimulation by self-assembled peptide-based vaccines. Peptides undergo self-assembly upon intra-muscular or subcutaneous vaccination, after which they can induce humoral and/or cellular immune responses to protect individuals against pathogens. Humoral immune responses arise once B-cells encounter antigens in secondary lymphoid organs, inducing their activation. Mechanistically, B-cell activation occurs upon binding of antigens to the B-cell receptor (BCR), resulting in the internalization of antigens via receptor-mediated endocytosis. These antigens are then processed, and antigenic peptide-loaded MHC II is displayed on the cell surface, allowing CD4+ helper T-cell binding. CD4+ helper T-cells further stimulate B-cells to undergo proliferation, immunoglobulin (Ig) class-switching, and differentiation into antigen-specific antibody-secreting plasma cells and memory B-cells. To induce CTL-mediated cellular immune responses, antigens need to be processed and presented by antigen-presenting cells (APCs), such as dendritic cells and macrophages. APCs take up the antigen by pinocytosis, phagocytosis, and receptor-mediated phagocytosis, cleave the antigen into smaller peptide fragments, and present these peptides on MHC. In the lymph nodes, extracellular antigenic peptides are presented on MHC II to CD4+ T-cells, whereas intracellular proteins, including viral and tumor-associated antigens, are presented on MHC I to CD8+ T-cells. A subset of APCs can also present extracellular antigenic peptides on MHC I in a process known as cross-presentation. Once activated, naïve CD8+ T-cells proliferate into CTLs to mediate antigen-specific cytotoxicity. A fraction of CD8+ T-cells become memory CD8+ T-cells to ensure long-term protection. Upon activation, naïve CD4+ T-cells differentiate into helper T-cells which secrete cytokines to support CTL expansion and survival along with B-cell proliferation and differentiation. Memory B- and T-cells persist in the body for a long time and mount an immediate and efficient antigen-specific immune response upon reinfection with the same pathogen.

The article "Supramolecular Self-Assembled Peptide-Based Vaccines: Current State and Future Perspectives" was published in 2020. Journal: Front Chem.

Additionally, non-peptidic compounds such as alkyls, amino acids, and metal ions have been used to form self-assembled peptide complexes with a wide variety of structures and functionalities (Sis and Webber, 2019). Alkyls, for instance, have been used as a hydrophobic tail to produce peptide amphiphiles (PAs) that undergo self-assembly via hydrophobic shielding (Sis and Webber, 2019). As a result, the nanostructure and other properties of self-assembled PAs can be controlled by switching their hydrophobic components (Qi et al., 2018). Choi et al. proved that the nanostructure of self-assembled amphiphilic Janus peptide dendrimers (JPDs) can be induced via a simple chemical bifurcation. Various JPDs were synthesized by varying the length of their hydrophilic and hydrophobic regions, and their self-assembly resulted in the formation of spherical/cylindrical micelles or bi-layered vesicles (Choi et al., 2019). PAs can also be made by conjugating peptides with functional polymers (Habibi et al., 2016). Chin et al. designed a muscle-inspired anisotropic actuator in the form of a hollow fibrous peptide-based hydrogel, in which VVVAAAEEE peptides were functionalized with a lysine-coupled bromoisobutyryl moiety to enable the grafting of thermo-responsive polymers via atom transfer radical polymerization (Chin et al., 2018). Recent studies also revealed that the nanostructure of self-assembled peptides can be reshaped in a controllable manner by incorporating metal ions (Sis and Webber, 2019). Knight et al. studied the effect of different metal ions on the morphological transformation of self-assembled PAs consisting of hexahistidine as a hydrophilic head and oligostyrene as a hydrophobic tail (Figure 1C). Interestingly, the presence of manganese(II) promoted the formation of multilamellar vesicles, while nickel(II) and cadmium(II) gave rise to micelle nanoparticles. In contrast, zinc(II), copper(II), and cobalt(II) led to agglomerated micelles (Knight et al., 2018).

Finally, there has been a growing interest in designing smart nanomaterials that initiate the assembly of molecular building blocks upon application of external stimuli such as enzymes, pH, heat, and light. This strategy can provide additional spatiotemporal control over the formation and structure of supramolecular peptides (Lampel, 2020). For instance, enzyme-instructed self-assembly (EISA) of peptides has recently been applied to allow assembly in complex biological systems (Wang et al., 2019). Li et al. synthesized several dipeptidic precursors, consisting of FF with various stereoisomers, in which N- and C-terminal peptide sequences are linked to 2-(naphthalen-2-yl)acetic acid and 2-(4-(2-aminoethoxy)-4-oxobutanamido)ethane-1-sulfonic acid, respectively. Molecular self-assembly (i.e., EISA) of these peptides is induced by carboxylesterase, which is present inside the cells and in the extracellular space of tissues. Using this approach, intracellular and intercellular peptide self-assembly could be achieved at different rates (Li et al., 2018). Additionally, some stimuli-responsive peptides, such as elastin-like polypeptides (ELPs), exhibit reversible transition behavior upon exposure to specific stimuli (Zhang et al., 2015; Saha et al., 2020). Dreher et al. prepared several ELP block copolymers (with varying molecular weights and block ratios) in a linear AB diblock architecture by homogeneously fusing an N-terminal hydrophilic ELP block to a C-terminal hydrophobic ELP block. They observed that copolymers with suitable diblock ratios are highly water-soluble at normal body temperature (37°C) and can self-assemble into spherical micelles at the tumor temperature (42°C). When the temperature was lowered again, the copolymers showed the inverse transition behavior (Dreher et al., 2008). Hassouneh et al. developed a theoretical model to explain the mechanism for this special reversible transition behavior of the copolymers (Hassouneh et al., 2015).

The article "Supramolecular Self-Assembled Peptide-Based Vaccines: Current State and Future Perspectives" was published in 2020. Journal: Front Chem.

## Application of Self-Assembled Peptides in Vaccine Design and Delivery

A wide variety of vaccines have been designed to stimulate the immune system to combat pathogens (e.g., bacteria, viruses) or tumors. In particular, vaccines aim to induce an adaptive immune response that leads to immunological memory, as illustrated in Figure 1D. There are two subdivisions of the adaptive immune system: the cell-mediated immune response, which is executed by cytotoxic T lymphocytes (CTLs) that can kill infected or cancerous cells, and the humoral immune response, which is mediated by activated B-cells that produce antibodies to neutralize extracellular pathogens (Molnar and Gair, 2015). Peptide-based vaccines generally require three major components—an antigen, an adjuvant, and a delivery vehicle—to generate efficient adaptive immune responses. When peptides are used as antigens, the conformation of the specific regions recognized by the immune system, known as epitopes, is particularly important for inducing humoral immunity. Specifically, B-cells need to bind epitopes in their native conformation to allow antibody binding. B-cell epitopes usually have α-helical, loop, and β-strand conformations that are generally integrated into vaccines as longer peptides to allow them to adopt their native conformation (Skwarczynski and Toth, 2016; Malonis et al., 2019). When designing vaccines, self-assembly of peptides can be utilized to ensure correct folding of antigenic epitopes. In vaccine applications where antibody affinity and titer are essential, self-assembling peptides that also have inherent CD4+ T-cell epitopes, such as those included in the Coil29 (QARILEADAEILRAYARILEAHAEILRAD) peptide, can be incorporated to induce strong follicular helper T-cell engagement that further promotes B-cell responses (Wu et al., 2020). Similar to CD4+ T-cell stimulation, the peptide sequence is more critical than the epitope conformation itself to induce CTL-mediated cellular immunity. Therefore, shorter peptides can be used to induce T-cell responses, as CD4+ T-cells recognize 12-16 amino acid long peptides presented by MHC II on antigen-presenting cells (APCs), while CD8+ T-cells bind to slightly shorter 8-10 amino acid long peptides displayed by MHC I (Skwarczynski and Toth, 2016; Malonis et al., 2019). Unlike attenuated pathogen-based vaccines, peptide-based vaccines generally incorporate adjuvants to boost the overall immune response to antigens and mimic the natural “danger signals” which follow infections. The choice of adjuvants depends on several factors such as immunogenicity and toxicity. Several studies have established that the adjuvanticity of self-assembled peptides is mediated via antigen presentation in an ordered and repetitive array that resembles pathogen-associated molecular patterns (PAMPs), resulting in strong immune responses mediated through Toll-like receptor (TLR)-inflammasome signaling pathways via TLR2 and TLR4 activation (Azmi et al., 2014; Negahdaripour et al., 2017; Tandon et al., 2018; Zottig et al., 2020). Additionally, self-assembling peptides may act as adjuvants themselves by forming an antigen depot, directing vaccines to APCs, and ultimately enhancing immune-cell priming (Grenfell et al., 2015; Acar et al., 2017; Negahdaripour et al., 2017).

### Self-Assembled Peptide-Based Vaccines for Cellular Immunity

Supramolecular self-assembling peptides can form excellent structures to induce cytotoxic immune responses, which is particularly important for cancer immunotherapy. For this purpose, peptide assemblies can function as a platform for safe and controlled delivery of antigens, adjuvants, immune cells and/or drugs (Table 1). For example, Wang et al. utilized a tumor-penetrating peptide Fmoc-KCRGDK-based hydrogel formulation to encapsulate a BRD4 inhibitor, a photothermal agent (indocyanine green), and autologous tumor cells. Upon laser irradiation, the personalized cancer vaccine released tumor-associated antigens. This process promoted DC maturation, T-cell infiltration, the formation of memory immune cells to prevent tumor relapse, and inhibited distant tumors (Wang T. et al., 2018). Interestingly, Xu et al. observed that the configuration and the number of lysine residues in the peptide are critical to enhance CTL response. They described a supramolecular NF-κB-activating nano-adjuvant hydrogel, synthesized by pH-triggered self-assembly of Ada-GFFYGKKK-NH2 peptide, for cancer immunotherapy. According to their findings, nano-adjuvants containing D-configured peptides and 3 lysine residues encapsulated antigens more efficiently through charge-charge interaction than 2 lysine residues, and as a result, generated more robust adaptive and innate immune responses than peptides with L-configuration (Xu et al., 2019). Yang et al. showed that a nanofibrous RADA16 peptide-based hydrogel scaffold encapsulating bone-marrow derived DCs, model antigen ovalbumin (OVA), and anti-PD-1 antibody recruited and stimulated endogenous and exogenous DCs. This process increased DC migration to the lymph nodes, driving a more robust antigen-specific immune response against EG7-OVA tumors (Yang et al., 2018). Furthermore, Wang et al. developed glutathione-responsive nanocomposites by co-assembling a positively charged cell-penetrating CWWRCRCRC peptide with a negatively charged protein such as ovalbumin (OVA) via electrostatic interactions. After being internalized by APCs, intracellular glutathione degraded the disulfide bonds of the peptide, inducing rapid release of the antigen into the cytoplasm, which was then cross-presented to induce potent CD8+ T-cell responses. When compared to free OVA, the peptide-based nanocomposites improved antigen uptake by DCs, promoted DC activation and maturation, and enhanced cellular as well as humoral immune responses (Wang K. et al., 2018). Overall, the use of self-assembled peptides as a delivery vehicle provides multiple benefits, including efficient cell and antigen loading, minimal loss of active components, as well as controlled and targeted release in the lymphoid organs (Zhang, 2017; Lee et al., 2019).

The article "Supramolecular Self-Assembled Peptide-Based Vaccines: Current State and Future Perspectives" was published in 2020. Journal: Front Chem.

**Table 1:** Summary of supramolecular peptide-based vaccines for cancer and infectious diseases.

**Peptide**	**Active ingredient**	**Features**	**Applications**	**References**
RADA16	Anti-PD-1 + DCs + OVA peptide	β-sheet-rich nanofibrous hydrogel	Delivery system for DC-based vaccine in EG7-OVA tumor model	Yang et al., 2018
K_2_(SL)_6_K_2_	STING agonist	Nanofibrous hydrogel with sustainable release properties	Delivery system in MOC_2_-E_6_E_7_ tumor model	Leach et al., 2018
Fmoc-KCRGDK	BRD4 inhibitor + indocyanine green + autologous tumor cells	Micellar hydrogel with tumor penetrating properties	Delivery system for postoperative cancer immunotherapy in 4T1 tumor model	Wang T. et al., 2018
Ac-I3SLKG-NH2	G(IIKK)3I-NH2	MMP-2 mediated enzyme responsive fibrillar hydrogels, sustained and targeted release properties	Delivery system for MMP-2 overexpressing HeLa tumor model	Chen et al., 2017
OVA_253−266_ peptide	OVA_253−266_ peptide conjugated with dialkyl lipid tail and 2 palmitic chains	Cylindrical micelles displaying epitopes at multiple valences with self-adjuvanting properties	Delivery system plus peptide tumor antigen in EG7-OVA tumor model	Black et al., 2012
OVA_254−267_-HBc (Hepatitis B core protein)	OVA_254−267_ peptide	Nanocage with controlled properties and high-density epitope display	Delivery system plus tumor antigen plus adjuvant for B16-OVA-Luc tumor model	Shan et al., 2019
Peptide-MHC/ANXA5	Peptide-MHC (pMHC)	Liposome	Antigen for B16-OVA tumor model	Mao et al., 2018
Ada-GFFYGKKK-NH2	OVA peptide	Nanofibrous hydrogel with NF-κB activating properties	Nano-adjuvant for B16-OVA cancer immunotherapy	Xu et al., 2019
Nap-GFFpY-OMe	OVA peptide	Nanofibrous hydrogel formed by phosphatase enzyme	Vaccine adjuvant for EG7-OVA tumor model	Wang et al., 2016
Q11 (QQKFQFQFEQQ)	Mucin 1 (MUC1) glycopeptide	Nanofibers, β-turn structure with self-adjuvanting properties	Delivery system plus adjuvant for MCF-7 tumor model	Huang et al., 2012
Ac-AAVVLLLW-COOH	OVA_250−264_ + HPV16 E7_43−57_	Nanostructure	TC-1 tumor model	Rad-Malekshahi et al., 2017
Cholesterol-aK-Cha-VAaWTLKAa-LEEKKGNYVVTDH	EGFRvIII + PADRE epitopes	Lipopeptide micelles with self-adjuvanting properties	Cellular and humoral immune response in B16-EGFRvIII tumor model	Chen et al., 2018
Coil29 (QARILEADAEILRAYARILEAHAEILRAD)	EGFRvIII, PADRE, SIINFEKL, PEPvIII	α-helical coiled-coiled peptide fiber	Induction of CD4+ T-cell, and CD8+ T-cell and B-cell response in mice	Wu et al., 2017
DEAP-DPPA-1	PD-L1 antagonist (^D^PPA-1) + peptide substrate of MMP-2 + indoleamine-dioxygenase inhibitor (NLG919)	Nanoparticle responding to dual stimuli for targeted delivery and controlled release	B16-F10 tumor model	Cheng et al., 2018
GE11 (EGFR ligand)	Acetylcholinesterase gene + Doxorubicin	Self-assembling peptide nanovesicle	Drug and gene delivery system targeted toward EGFR expressing cancer	Liang et al., 2016
S4-8Q (QAEPDRAHYNIVTFCCKCD conjugated to a 4-arm star polymer)	8Q (HPV-16 E7 epitope)	Dendrimers with self-adjuvanting properties	TC-1 tumor model	Liu et al., 2013; Liu et al., 2015
Nap-GFFY-NMe	DNA encoding gp145	Nanofibrous hydrogel	Strong cellular and humoral immune response for HIV treatment and prevention	Tian et al., 2014
EAK16-II	SL9 (HIV specific CTL epitope) + TL13 (CD4+ T-cell epitope) + R848 (TLR7/8 agonists) + DCs	β-sheet-rich nanofibers	Delivery system for HIV-1 vaccine	Ding et al., 2016
p41	p41 peptide (analog derived from HCV protein NS5A)	α-helical nanocomplexes	HIV and HCV co-inhibition	Zhang et al., 2013
P6HRC1	HRC1 (B-cell epitope from S-protein)	Coiled-coil polypeptide nanoparticles	Coronavirus mediated SARS (severe acute respiratory syndrome) infection	Pimentel et al., 2009
KFE8	EIII (West Nile Virus envelope protein domain)	β-sheet-rich nanofibrous hydrogel with self-adjuvanting properties	West Nile virus vaccine	Friedrich et al., 2016
Pentamer and trimer sequence	PspA and CbpA (CTL epitopes) + PhtD and PiuA (helper T-cell epitopes) + DTD (universal T-helper)	5-stranded + 3-stranded coiled-coils nanoparticle scaffold with self-adjuvanting properties	*Streptococcus pneumoniae* vaccine	Dorosti et al., 2019
J8 B-cell epitope: (SREAKKQVEKAL)	J8 conjugated with dialkyl hydrophobic moiety (diC16)	Cylindrical micelles with self-adjuvanting properties	Group A *Streptococcus pyogenes* vaccine	Trent et al., 2015
MAX1	Inherently antibacterial	β-hairpin-rich hydrogel	Broad spectrum bacterial resistance to gram-positive and gram-negative bacteria	Salick et al., 2007
Fmoc-F_2_	Silver nanoparticles	Macroscopic hydrogels	Anti-bacterial wound dressing	Paladini et al., 2013
Phage-VS-LK	Sap2 (VS) + Hsp90 (LK) peptides	Nanofiber	*Candida albicans* detection via ELISA and vaccine	Wang T. et al., 2018
Cholesterol-G3R6TAT	Inherently antimicrobial	Nanoparticles	*Cryptococcus neoformans-*induced mengitis	Wang et al., 2010
Q11	NANP_3_ (circumsporozoite protein epitope)	β-sheet-rich nanofibers	*P. falciparum* vaccine for malaria	Rudra et al., 2012

Apart from acting as a delivery vehicle, self-assembling peptides can also serve as an antigen source themselves to induce cellular immunity. For example, Black et al. developed cancer vaccines consisting of self-assembling tumor antigen peptides with enhanced immunogenicity. Conjugating a synthetic lipid tail with two palmitic residues to an OVA-derived peptide containing a CTL epitope initiated the self-assembly of PAs into cylindrical micelles, resulting in multivalent epitope presentation. These micelles were internalized by APCs, likely due to the fusion of their hydrophobic tails with the cell membrane, leading to CTL activation in absence of additional adjuvants. Additionally, these cylindrical micelles act as antigen depots, thereby protecting the peptides from degradation and prolonging antigen exposure to the APCs. Improved *in vivo* protection was observed against OVA-expressing tumor cells after immunization with the diC16-OVA micelles compared to free OVA peptide formulated with incomplete Freund's adjuvant (Black et al., 2012). Xing et al. developed injectable, peptide-based supramolecular hydrogels by co-assembling poly-L-lysine (PLL) and FF dipeptide via an electrostatic coupling. Fmoc-FF/PLL-SH hydrogels have a nanofibrous structure with α-helical conformation which resembles natural fimbrial antigens, thereby acting as an adjuvant. When injected around a tumor, the hydrogels activated T-cell responses and efficiently suppressed tumor growth without the addition of other adjuvants or antigens. In this case, the tumor cells themselves act as the source of antigen to stimulate the immune response (Xing et al., 2017). Self-assembly can also be used to incorporate longer peptides containing multiple epitopes to ensure optimal APC stimulation, increase the magnitude of CTL response, and simultaneously promote helper T-cell activity (Lynn et al., 2020). Overall, peptide-based self-assembly can induce robust cellular immune responses by serving as a durable source of antigen that allows easy uptake and processing by APCs, providing multiple epitopes, and conferring self-adjuvanticity to the vaccine.

The article "Supramolecular Self-Assembled Peptide-Based Vaccines: Current State and Future Perspectives" was published in 2020. Journal: Front Chem.

### Self-Assembled Peptide-Based Vaccines for Humoral Immunity

Robust humoral immune responses are essential to treat infectious diseases. For this purpose, self-assembly designs have included approaches such as flanking the antigen with a self-assembling peptide sequence to display the secondary structure of the antigen, presenting antigens in a highly ordered and repetitive form, and optimizing the distance between repeated epitopes for optimal B-cell receptor (BCR) engagement (Raman et al., 2006; Black et al., 2010; Babapoor et al., 2011; Trent et al., 2015; Skwarczynski et al., 2020). Self-assembling supramolecular peptides can serve as a delivery scaffold to present antigenic peptides, and they can simultaneously possess self-adjuvanting characteristics to induce B-cell responses. For instance, Grenfell et al. exploited RADA4 peptide-based hydrogels that self-assembled into hydrated nanofibers after injection into the tissue to form a gel matrix depot, to deliver a recombinant antigen for the hepatitis B virus. This system elicited enhanced adjuvant-free humoral and cellular responses when compared to the antigen delivered with aluminum hydroxide (alum) and complete Freund's adjuvant. The authors credited the slow release of antigen from the depot to have improved the activation of APCs and prolonged immunostimulation (Grenfell et al., 2015). In a different study, Tian et al. utilized a supramolecular hydrogel-based nanovector comprised of Nap-GFFY-NMe (naphthylacetic acid-modified tetrapeptide GFFY with C-terminal methyl amide group), using an EISA approach to encapsulate a DNA sequence encoding gp145, an envelope glycoprotein of the human immunodeficiency virus (HIV). Alkaline phosphatase triggered self-assembly of the peptide, leading to formation of nanofibrous hydrogels. The strong cellular and humoral immune responses were attributed to the ability of left-handed structure of nanofibers to effectively condense DNA and prevent it from degradation, thus enhancing DNA transfection and gene expression in cells (Tian et al., 2014).

The article "Supramolecular Self-Assembled Peptide-Based Vaccines: Current State and Future Perspectives" was published in 2020. Journal: Front Chem.

Self-assembling peptides can also be an antigen source to induce humoral immunity. For instance, Kaba et al. utilized a self-assembling peptide-based nanoparticle platform to present repeated immunodominant B-cell circumsporozoite peptide epitope (DPPPPNPN)_2_D of the malarial parasite. The polypeptide consisted of two oligomerization domains—a *de novo* trimeric coiled-coil domain and a pentameric coiled-coil domain—which were fused together with flexible diglycine residues. The self-assembled nanoparticles, containing multiple coiled-coil domains, displayed the B-cell peptide epitope in a highly ordered and repetitive array, thereby triggering robust helper T-cell-dependent and long-lasting antibody responses with higher avidity and titer (Kaba et al., 2009). Pimentel et al. utilized a similar polypeptide-based self-assembling nanoparticle platform to display the C-terminal heptad repeat region (HRC) of the SARS-CoV S-protein in its native α-helical trimeric coiled-coil conformation. These nanoparticles not only maintained this conformational integrity, but also provided repetitive presentation of the B-cell epitope and displayed icosahedral symmetry that resembled viral protein capsids. The SARS-CoV vaccine evoked conformation-specific neutralizing antibodies against the B-cell epitope without additional adjuvants (Pimentel et al., 2009). A potent peptide-based vaccine against *Streptococcus pneumoniae* was proposed by Dorosti et al., who incorporated CTL epitopes such as pneumococcal surface protein A (PspA) and choline-binding protein A (CbpA), helper T-cell epitopes such as pneumococcal histidine triad protein D (PhtD) and a lipoprotein from pneumococcal iron ABC transporter (PiuA) and universal helper T-cell epitopes like diphtheria toxoids on a coiled-coil self-assembling interface. The designed vaccine was predicted to exhibit stronger immunogenic responses compared to an analogous epitope-based vaccine (Dorosti et al., 2019). In addition, Rudra et al. developed a peptide-based vaccine to prevent malaria by combining self-assembling β-sheet peptides with epitopes of protozoan parasite *P. falciparum* (Rudra et al., 2012). In another example, Trent et al. designed a self-adjuvanting peptide-based vaccine for group A streptococcus (GAS). When the J8 antigenic peptide of the GAS-M protein is taken out of its native protein environment, its α-helical structure is lost, and as a result, it adopts a random conformation in the solution. The addition of two C16 alkyl chains at the N terminus of the J8 peptide triggered its self-assembly into cylindrical micelles, and reinforced α-helicity of the antigen, which subsequently induced a strong B-cell response in mice. Since the hierarchical micellar structure kept thousands of peptides in close proximity, it conferred potent adjuvanticity while maintaining the native antigen conformation at the injection site. In addition, the micellar structure increased the local antigen concentration available to immune cells in comparison to free peptide, which quickly diffused away from the injection site (Trent et al., 2015). Taken together, these studies have demonstrated that self-assembled peptides can efficiently induce humoral immune responses through the display of secondary structures, thereby maintaining the conformational integrity of epitopes. Furthermore, these self-assembly platforms offer a highly ordered and multivalent display of relevant antigens, resulting in efficient stimulation and proliferation of B-cells, and their subsequent differentiation into antibody-secreting plasma cells. Inclusion of helper T-cell epitopes further enhances vaccine efficacy by imparting long-lasting B-cell immunity.

The article "Supramolecular Self-Assembled Peptide-Based Vaccines: Current State and Future Perspectives" was published in 2020. Journal: Front Chem.

## Challenges and Future Perspectives

Despite the great potential of self-assembled supramolecular peptides for vaccine design and engineering, many challenges still persist. Compared to conventional vaccines containing live-attenuated or inactivated pathogens (viruses, bacteria, etc.), most peptide-based vaccines induce a weak immune response (Malonis et al., 2019). The use of adjuvants can overcome this obstacle, and deepen our understanding of their mechanism of action and their safety (Skwarczynski and Toth, 2016). Additionally, maintaining the stability and efficacy of peptide-based vaccines in complex biological environments remain challenging. For instance, their rapid enzymatic degradation and structural integrity in the body is a major limiting factor (Kim et al., 2019). Self-assembled peptides must exhibit improved stability when interfacing with biological barriers (e.g., pH, enzymes) that are encountered upon administration in tissues (Eskandari et al., 2017). Rational systematic design of the supramolecular peptide structure to include covalent cross-linking—or via improved intermolecular interactions such as hydrogen bonding, π-π stacking, and hydrophobic interactions—may augment their resilience and mechanical stability (Khalily et al., 2015; Li et al., 2019). The development of supramolecular self-assembled peptide-based vaccines is hindered by our limited understanding of the interface between self-assembled nanostructures and immune cells. In-depth investigation of the interactions between the self-assembled structures and the receptors on human immune cells, their uptake by APCs, as well as their effect on DC maturation, B-cell and T-cell priming, and cytokine profile, is needed (Zhao et al., 2017). Challenges exist in translating the ease in design and small-scale synthesis of supramolecular peptides to an industrial scale. Furthermore, advanced engineering of supramolecular assembly (e.g., cell-penetrating peptides) may target intracellular vaccine delivery more precisely, ultimately enhancing antigen uptake, promoting endosomal escape and cross-presentation by APCs, which are critical steps in inducing a robust cellular immune response (Yang et al., 2019). Existing technologies such as machine learning, bioinformatics, and computational modeling can potentially be leveraged for the macromolecular engineering of immunostimulatory peptide assemblies with improved vaccine immunogenicity, efficacy, and safety (Kim et al., 2019). Moving forward, biologically inspired supramolecular peptides, an excellent and sparsely explored class of materials, could be further exploited in designing the next generation of vaccines that are effective, safe, affordable, and accessible to everyone. Despite their importance and great potential, self-assembled peptide-based vaccines do require further investigation and validation prior to regulatory approval and clinical use.

## Author Contributions

The manuscript was written and edited with contribution from all authors. All authors have given approval to the final version of the manuscript.

## Conflict of Interest

KB is currently a student at Northeastern University and employed by Moderna Inc. However, Moderna Inc. was not involved in the writing of this review article or the decision to submit it for publication. The remaining authors declare that the research was conducted in the absence of any commercial or financial relationships that could be construed as a potential conflict of interest.
